The article "Neuroprotective Effects of Hesperetin in Regulating Microglia Polarization after Ischemic Stroke by Inhibiting TLR4/NF-κB Pathway" was published in 2021. Journal: J Healthc Eng.

# Neuroprotective Effects of Hesperetin in Regulating Microglia Polarization after Ischemic Stroke by Inhibiting TLR4/NF-*κ*B Pathway

**DOI:** 10.1155/2021/9938874

**Published:** 2021-12-17

**Authors:** Jiawen Zhang, Hao Jiang, Fang Wu, Xiaofei Chi, Yu Pang, Hongwei Jin, Yuyang Sun, Shicun Zhang

**Affiliations:** ^1^Department of Neurology Four Ward, The Second Affiliated Hospital of Qiqihar Medical University, Qiqihar 161000, China; ^2^The Fifth Affiliated Hospital of Harbin Medical University, Qiqihar 161000, China; ^3^Division of Liver Disease, Qiqihar Seventh Hospital, Qiqihar 161000, China

## Abstract

This study aimed to explore the influence of hesperidin on the polarization of microglia to clarify the key mechanism of regulating the polarization of M2 microglia. C57BL/6 mice were randomly divided into middle cerebral artery occlusion model group (MCAO group), MCAO + hesperidin treatment group (MCAO + hesperidin group), and sham group (sham operation group). The mice were assessed with neurological scores for their functional status. 2,3,5-Triphenyltetrazole chloride (TTC) was used to determine the volume of cerebral infarction. Hematoxylin and eosin (H&E) staining was performed to detect brain loss. The system with 1% O_2_, 5% CO_2_, and 92% N_2_ was applied to establish BV2 in vitro model induced by MCAO. TNF-*α*, IL-1*β*, TGF-*β*, and IL-10 levels of cytokines in the supernatant were detected by ELISA. RT-qPCR was used to detect mRNA levels of M1 iNOS, CD11b, CD32, and CD86, and mRNA levels of M2 CD206, Arg-1, and TGF-*β*. The Iba-1, iNOS, and Arg-1 of microglia and protein levels of TLR4 and p-NF-*κ*B related to the pathway were detected by Western blot. After treatment with hesperidin, BV2 cells induced by MCAO in vitro can reduce the proinflammatory cytokines of TNF-*α* and IL-1*β* significantly, further upregulating anti-inflammatory cytokines of TGF-*β*, IL-10 while inhibiting TLR4 and p-NF-*κ*B expression. The MCAO-induced BV2 cells treated by TLR-4 inhibitor TAK-242 and NF-*κ*B inhibitor BAY 11-7082 had similar polarization effects to those treated with hesperidin. This study found that hesperetin gavage treatment can improve the neurological deficit and regulate the polarization of microglia in MCAO mice. In vitro experiments further verified that hesperidin plays a neuroprotective role by inhibiting the TLR4-NF-*κ*B pathway, thus providing new targets and strategies for neuroprotection and nerve repair after ischemic stroke.

## 1. Introduction

Ischemic stroke is the third most common cause of human death in modern society, which may be caused by a combination of many factors. A preferred effective treatment for ischemic stroke is intravenous administration of tissue plasminogen activator (tPA), which can only benefit patients who receive the treatment within a time window of 4.5 h after stroke. For patients who miss the optimal time for thrombolysis, there is no safe and effective treatment, with high mortality. For the surviving patients, most of them have neurological disorders such as limb and language [1]. Recent studies have found that inflammation and immune response after stroke can aggravate nerve cell injury, and overactivated inflammatory cells and cytokines cause a local chronic inflammatory response, which is not conducive to repairing nerve cells [2–4].

Studies have shown that microglia in the adult brain are derived very early from primitive myeloid progenitor cells in the yolk sac [5]. Known as the innate immune cells of the brain, it plays an important role in the development of the central nervous system, the formation of the synapsis, and immune balance. In the absence of stress, microglia are involved in the development and pruning of synapsis [6]. Under pathological conditions, microglia are also involved in the inflammatory response at all stages in developing many diseases of the nervous system, including stroke, Parkinson's disease, and Alzheimer's disease [7–11]. After ischemic stroke, microglia can be driven to a “classic activated” proinflammatory (M1) phenotype and a “selective activated” anti-inflammatory (M2) phenotype. Studies have shown that the inflammatory factors of M1 phenotype can be upregulated. For example, proinflammatory cytokines, such as interleukin (IL)-1*β*, IL-2, and IFN-*γ*, CXC motif chemokine ligand 9 (CXCL9), CXCL10, inducible nitric oxide synthase (iNOS), and cyclooxygenase 2 (COX-2), can aggravate symptoms after stroke. Selective inhibition of minocycline on M1 microglia can significantly improve ischemic injury by reducing inflammatory response [12]. Furthermore, some studies have shown that, after stroke, M2 population has neuroprotective effects [3, 13–15]. M2 microglia activated after the ischemic injury can express high levels of arginase-1 (Arg-1), interleukin-10 (IL-10), transforming growth factor *β* (TGF-*β*), and insulin-like growth factor-1 (IGF-1). M2 phenotypes can prolong neuronal survival and inhibit brain injury [10, 16]. However, microglial cells activated after cerebral ischemia show only a transient M2 phenotype and subsequently a deleterious M1 phenotype [13].

Hesperidin (30,5,7-trihydroxy-4-methoxyhuangketone) is a member of the flavanone subclass of flavonoids found in citrus fruits, such as oranges and grapefruit. Previous studies have shown that hesperidin has significant antioxidant, anti-inflammatory, antiapoptotic, and antitumor effects [17–20]. Moreover, it inhibits inflammation in various cells by regulating extracellular signal-regulated kinase (ERK)1/2, p38 mitogen-activated protein kinase (MAPK) signaling pathways [21]. Hesperetin has been reported to protect the AD rat model against memory impairment during elevated oxygen stress [22]. There are few studies on ischemic stroke. This study aimed to explore the regulation of hesperidin on the polarization of microglia after cerebral ischemia, as well as its mechanism, so as to provide new targets and strategies for neuroprotection and nerve repair after ischemic stroke.

## 2. Methods

### 2.1. Middle Cerebral Artery Occlusion (MCAO) Model

A total of 30 male C57BL/6 strain mice were purchased from Nanjing Model Animal Research Institute. The mice were 10–12 weeks old and about 22–26 g. They were acclimatized for 3–5 d at room temperature 22–25°C in SPF class animal rooms before the experiment. The mice were randomly divided into MCAO group, MCAO + hesperidin group, and sham group, with ten in each group. After a 3.5% pentobarbital anesthesia, referring to Hu et al., right MCAO was induced, and the blood flow was restored 60 min after transient focal cerebral ischemia. The rectal temperature was maintained at 37.0 ± 0.5°C with a temperature-controlled heating pad throughout the operation. The hesperidin suspension was prepared by dissolving hesperidin (≥95%, Sigma-Aldrich, W431300) in 0.5% carboxymethyl cellulose solution. The MCAO + hesperidin group was given fresh hesperidin suspension prepared daily after MCAO operation. 30 mg/kg of constant volume was administered once a day for 7 d. All sham-operated animals received the same surgical protocol except MCAO. The MCAO and sham groups were given 0.5% carboxymethyl cellulose liquid of the same volume, which contained only a medium solution (0.5% carboxymethyl cellulose). According to the Longa scoring method, neurological deficit score was evaluated on the 1st, 3rd, 5th, and 7th d after surgery. The criteria were as follows: 0, normal, no neurological deficit; 1, mild neurological deficit, cannot fully extend the left front claw; 2, moderate neurological deficit, turn left; 3, severe neurological deficits, fall to the left; 4, no spontaneous movement, low levels of consciousness; 5, death; only animals with scores of 1 to 4 were used in this experiment [23]. After 14 days of operation, each group of mice was anesthetized with apical blood and then perfused with precooled PBS, and the fresh brain tissue of the mice was removed for a follow-up test. All animal experiments were carried out in accordance with the guidelines for Guidelines for the Care and Use of Laboratory Animals (NIH, No. 85-23, 1996) and were approved by the Ethics Committee of the Second Affiliated Hospital of Qiqihar Medical College. All surgery and subsequent analyses were performed by blind method.

### 2.2. Analysis on Volume of Cerebral Infarction and Brain Loss

The volume of cerebral infarction was determined by 2-,3-,5-triphenyl tetrazolium chloride (TTC) [24]. H&E staining was performed to detect brain loss, which was measured by subtracting the nonpathogenic area of the ipsilateral hemisphere from the area of the contralateral hemisphere. The volume of tissue loss was calculated from the lesion area of six parts. Image J (1.52a) software was used for calculation and analysis.

### 2.3. Cell Culture

Under normal conditions (20% O_2_, 5% CO_2_), BV2 cells were cultured with conventional high glucose DMEM in a 37°C incubator. Then, they were divided into normal group, MCAO group, MCAO + hesperidin (100 *μ*M) group, MCAO + TAK-242 group, and MCAO + BAY group. After growing to 50% density, MCAO was induced by transferring BV2 cells into DMEM without glucose and serum (Life Sciences, Inc., USA) and N_2_ was inflated for 5 min prior to administration. The dishes were then placed in an incubator at 37°C (containing 1% O_2_, 5% CO_2_ and 92% N_2_) in the presence or absence of hesperidin for 24 h before the medium was changed. After processing, the medium containing hesperidin was removed, replaced with the normal full medium. TAK242 (2 *μ*M; Sigma-Aldrich, 243984) or BAY 11-7082 (15 *μ*M; Sigma-Aldrich, B5556) was adopted for specific inhibition of TLR4 and NF-*κ*B. All chemicals/drugs were sterile and incubated at 5% CO_2_ and 37°C for 24 h.

### 2.4. RT-qPCR

About 5 mg total RNA was extracted from the microglial cell line or brain tissue in the affected area with Trizol (Qiagen, Hilden, Germany). And then, Superscript III First-Strand Synthesis SuperMix (Invitrogen, Carlsbad, CA, US) was applied to transcript RNA as cDNA. cDNA and SYBR GREEN FAST mastermix (Qiagen) was adopted for RT-qPCR, as follows: at 95°C for 3 min, at 95°C for 30 min, at 55°C for 1 min, for 40 cycles. Each sample was provided with three secondary holes. All primers used in the RT-qPCR were purchased from Sangon Biological Co., Ltd. Data were collected from the RT-qPCR system (Bio-Rad, Hercules, CA, USA), with GAPDH as an internal control. The relative quantitative value of each gene was calculated with the comparative cycle threshold method. All experiments were repeated three times, and the target gene was calculated by 2^−∆∆Ct^. See Table 1 for primer sequences.

### 2.5. Western Blot

Brain samples or cultured cells were sonicated in precooled RIPA lysate (Beyotime) for 1 min, and 12,000 g was taken to centrifuge for 10 min at 4°C, and the supernatant was stored at −80°C. Protein concentration in the sample was determined with the BCA Protein Assay Kit (Beyotime). The extracted proteins were separated by 10% SDS-polyacrylamide gel electrophoresis and transferred to PVDF (Millipore, Bedford, MA, USA). The membrane was sealed in a TBST buffer containing 5% skimmed milk for 1 h and incubated overnight at 4°C with the following primary antibodies: anti-mouse-iba-1 (sc-32725, 1 : 1000), anti-mouse-TLR4 (sc-16240, 1 : 1000), anti-mouse-p-NF-*κ*B (sc-136548, 1 : 1000), anti-mouse-*β*-actin (sc-47778, 1 : 1000), anti-mouse-iNOS (BD-610329, 1 : 1000), and anti-mouse- Arg-1 (sc-F0915, 1 : 1000). The membrane was then washed with TBST and incubated with horseradish peroxidase-labeled goat anti-mouse IgG (Biyuntian, A0216, 1 : 5000) and secondary antibody at room temperature for 1 h. The protein bands were detected with an enhanced chemiluminescence detection system (Bio-Rad, Hercules, CA, USA) and quantified with Image Lab software (Bio-Rad).

### 2.6. ELISA

For measuring the levels of IL-1*β*, IL-10, TNF*α*, and TGF-*β* in the cell medium, the supernatants of BV2 cells in the medium under different treatment conditions were collected, and 300 g was taken to centrifuge for 10 min to remove the precipitation. According to the corresponding instructions of the ELISA kit (UNOCI Biotechnology Co., Ltd; EK201B/3; EK210/3; EK282/3; EK981), the test was operated, with the sensitivity of 1.45 pg/ml, 4.8 pg/ml, 1.63 pg/ml, and 3.36 pg/ml, respectively. An enzyme marker was adopted for double wavelength detection within 30 min, to determine the maximum absorption wavelength as 450 nm. The standard curve was generated by regression fitting with the standard concentration as the abscissa and OD value as the ordinate, and the fitting equation was generated. The corresponding cytokine concentration was calculated according to the OD value.

### 2.7. Statistical Analysis

The statistical analysis was conducted on all data with SPSS 17.0 software, and the measurement data were expressed as mean ± standard deviation (*x* ± sd) data. *T*-test was used to compare the neurological function score, cerebral infarction volume, and brain loss volume. The relative expressions of protein, mRNA relative level, cytokine level, and so on were compared by ANOVA and Bonferroni method. All experiments were repeated at least 3 times. *P* < 0.05 was considered statistically significant.

## 3. Results

### 3.1. Hesperidin Can Improve the Neural Function Defect with a Protective Role in MCAO Mice

The ischemic stroke was simulated with a model of middle cerebral artery occlusion, and the patients were given 30 mg/kg hesperidin carboxymethyl cellulose solution by gavage immediately after surgery, repeated every day. For seven days, the control group was given 0.5% carboxymethyl cellulose solution after surgery. The neurological deficit symptoms of mice were dynamically evaluated every other day, and the neurological deficit score was recorded. The results showed that the neurological deficit symptoms in the MCAO + hesperidin group were significantly reduced compared with those in the MCAO group (Figure 1(a)). And over time, there has been a trend of gradual recovery of nerve function. Brain tissue was taken 7 days after MCAO to evaluate cerebral infarction volume and brain loss volume. It was found that the volume of cerebral infarction and brain loss after treatment with hesperidin was significantly lower than that in the model group (*P* < 0.01; *P* < 0.001, as shown in Figures 1(b) and 1(c)).

### 3.2. Hesperidin Can Regulate the Polarization of Microglia Cells in Brain of MCAO Mice

For further study of the polarization state of microglial cells in MCAO mice, we used fluorescence RT-qPCR to detect the mRNA levels of M1 microglia and M2 microglia-related cytokines and surface molecules in infarct lateral brain tissue and found that the mRNA levels of the molecules representing M1 microglia, such as iNOS, CD11b, CD32, and CD86, in the infarct side brain tissues of MCAO group were significantly higher than those of the MCAO + hesperidin group and sham group. It indicated that M1 microglia are significantly activated after MCAO, and the mRNA expression of M1 microglia-related molecules can be significantly inhibited by hesperidin therapy (*P* < 0.001; *P* < 0.001; *P* < 0.001; *P* < 0.001), as shown in Figures 2(a)–2(d). The protein level results also validated the overactivation of microglia in the lateral brain tissue of post-MCAO infarction. After treatment with hesperidin, the microglia and the molecular Iba-1 and iNOS of M1 microglia were significantly inhibited, as shown in Figures 3(a) and 3(b) (*P* < 0.01; *P* < 0.05). Instead, molecules of M2 microglia were significantly inhibited after MCAO (*P* < 0.05). As shown in Figures 2(e)–2(h), the mRNA levels of M2 microglia-related molecular CD206, Arg-1, TGF-*β* and Ym1/2 in the MCAO group were higher than those in the sham group but significantly lower than those in the MCAO + hesperidin group (*P* < 0.001; *P* < 0.001; *P* < 0.001; *P* < 0.001). WB results were consistent with mRNA results (Figures 3(a) and 3(b)), demonstrating that the therapy given to the MCAO + hesperidin group can inhibit the activation of proinflammatory M1 microglia, upregulating the polarization of anti-inflammatory M2 microglia.

### 3.3. Hesperidin Can Inhibit TLR4 and p-NF-*κ*B Expression in MCAO Mice

To further clarify the mechanism of how hesperidin regulates the polarization of microglia, we used Western blot to detect TLR4 and p-NF-*κ*B expression in the lateral cerebral tissue of infarcted mice 7 days after surgery, as shown in Figures 3(a) and 3(c). TLR4 and P-NF-*κ*B expression in infarct side brain tissue of mice in MCAO group were significantly higher than those in sham group (*P* < 0.001). Both TLR4 and p-NF-*κ*B were significantly inhibited after treatment with hesperidin, and the difference was statistically significant, *P* < 0.001.

### 3.4. Hesperetin Can Regulate Cytokine Changes in MCAO-Induced BV2 Cells

To explore the mechanism of hesperidin regulating microglia, we have established a BV2 MCAO induction system in vitro and found that, under MCAO conditions, the levels of proinflammatory cytokines TNF-*α* and IL-1*β* and anti-inflammatory cytokines TGF-*β* and IL-10 in the supernatant of BV2 cells were significantly increased compared with those of normal cultured cells, as shown in Figures 4(a)–4(d) (*P* < 0.001). Under hypoxic conditions after adding hesperidin, the proinflammatory cytokines were significantly decreased, while the anti-inflammatory cytokines were further upregulated. In animal experiments, upregulation of p-NF-*κ*B and TLR-4 after MCAO was found. To verify this mechanism, we treated MCAO-induced BV2 cells in vitro with TLR-4 inhibitor TAK-242 and NF-*κ*B inhibitor BAY 11-7082, respectively. It turned out that, after treatment with these two inhibitors, the upregulation of proinflammatory cytokines was inhibited under MCAO conditions, while anti-inflammatory cytokines were further upregulated, which were basically the same as those of the MCAO + hesperidin group, as shown in Figures 4(a)–4(d), except for IL-1*β*. There was no statistical difference between the other cytokines and the MCAO + hesperidin group.

### 3.5. Hesperidin Can Regulate Phenotypic Changes of BV2 Cells Induced by MCAO through TLR4-NF-*κ*B Pathway

The expression of iBA-1 and iNOS in BV2 cells induced by MCAO in vitro was significantly higher than that in the MCAO + hesperidin group, while the expression of ArG-1 was significantly lower than that in the MCAO + hesperidin group. It indicated that hesperidin can inhibit the expression of proinflammatory type and upregulate the expression of anti-inflammatory type in MCAO-induced BV2 cells (Figures 5(a) and 5(b)). Then, MCAO-induced BV2 cells were treated with TLR-4 inhibitor TAK-242 and NF-*κ*B inhibitor BAY 11-7082. We found that both inhibitors can inhibit the expression of proinflammatory and upregulate the expression of anti-inflammatory type, similar to the effect of hesperidin (Figures 5(a) and 5(b)). In addition, the expression levels of TLR-4 and P-NF-*κ*B in BV2 cells in MCAO group were significantly lower than those in MCAO + hesperidin group, MCAO + TAK-242 group, and MCAO + BAY group. The expression levels of TLR-4 and P-NF-*κ*B in MCAO + hesperidin group were consistent with those in MCAO + TLR-4 group and MCAO + NF-*κ*B group (Figures 5(a), 5(c), and 5(d)), suggesting that hesperidin regulates the phenotypic changes of MCAO-induced BV2 cells through TLR4-NF-*κ*B pathways.

## 4. Discussion

Ischemic stroke is the third leading cause of human death, accounting for 9% of the world's deaths, with high morbidity, mortality, and disability. Recently, studies have found that poststroke inflammation and immune responses exacerbate neuronal injury, which runs through every stage of ischemic stroke, varying degrees of activation from the early stages of destructive events to the later stages of brain tissue repair and vascular regeneration [2–4]. In further studies of these findings, postischemic stroke autopsy results and animal experiments strongly demonstrated the significant role of poststroke inflammation [25–29]. After ischemic stroke occurs, microglia can be driven to a “classic activated” proinflammatory (M1) phenotype and a “selective activated” anti-inflammatory (M2) phenotype. M1 microglia can secrete a variety of cytokines, causing inflammatory response, which is not conducive to the recovery of injured nerve tissue, while M2 microglia have neuroprotective effects.

In this study, we found that the mRNA level and iNOS protein expression of M1 microglia-related molecules increased significantly in infarcted lateral brain tissue of MCAO of mice, while the mRNA level and Arg-1 protein level of type M2 related molecules increased after hesperidin treatment. The neurological deficit symptoms of mice improved and the activation level of M1 cells decreased, which is consistent with the study of Kobayashi et al. [12]. The production of inflammatory cytokines, such as TNF, IL-1, and IL-6, is one of the most important capabilities of microglia/macrophages. On the one hand, proinflammatory cytokines lead to neuronal death through direct or indirect pathways, such as necrosis, apoptosis, and pyrophosphate processes mediated by inflammatory corpuscles and cysteinase family proteins [30, 31]. On the other hand, proinflammatory cytokines can regulate the phagocytic activity of microglia/macrophages. Studies have shown that TNF-*α* downregulates the expression of microglia CD36, resulting in the loss of phagocytic capacity of microglia to phagocytosis of hematoma after intracerebral hemorrhage [32]. Similarly, higher TNF-*α* expression levels were found to be consistent with higher microglial phagocytosis after ischemic stroke [25].

Protective effects of M2 phenotypes are mediated mainly by the ability to engulf debris and promote repair and regeneration of brain tissue after cerebral ischemia [33]. The clearance of apoptotic and necrotic cells by microglia is particularly important for maintaining central nervous system homeostasis in pathological conditions. Removing injured neurons not only prevents secondary inflammatory response, but also makes room for new neurons and reconstruct the balance of the body, which is beneficial to the survival of new neurons [34, 35]. Moreover, the activation of microglia contributes to the abnormal migration of newborn neurons and may play a beneficial role in the regulation of neurogenesis through the production of neurotrophic mediators such as IGF-1 and TGF-*β* [36, 37]. Other markers M2 microglia, such as Ym1 and Arg-1, can prevent degradation of extracellular matrix components [38]. In addition, microglial activation can promote regeneration by removing disabled synapses, facilitating the formation of functional synapses [39–41].

Recently, studies on hesperidin in microglia regulation have found that hesperidin can strongly inhibit nitric oxide production and inducible nitric oxide synthase expression in LPS stimulated BV-2 microglia. The secretion of inflammatory cytokines including interleukin IL-1b and IL-6 can also be significantly reduced by hesperidin [42]. Moreover, hesperidin can downregulate the phosphorylation of extracellular signal-regulated kinase (ERK)1/2 and p38 mitogen-activated protein kinases, with an anti-inflammatory role. Furthermore, hesperidin can inhibit the activation of astrocytes and microglia, which participates in TLR4/NF-*κ*B mediated signaling pathways in the brain of LPS attacked mice [43].

TLR is a family of innate immune receptors that play an important role in regulating inflammation and participate in stroke-induced neuroinflammation, and several studies have confirmed that TLR is an important therapeutic target for stroke treatment [44]. In a study of TLR4-deficient mice, Sansing et al. found that the TLR4 signaling pathway leads to inflammation and damage around post-ICH hematomas [45] and confirmed that TLR4 activation on microglia is triggered by heme via the MyD88/TRIF signaling pathway [46]. TLR4 antagonists TAK242 reduce these deleterious effects of stroke TLR4 signal transduction [47]. Furthermore, TLR2/TLR4 heterodimer formation may result in severe neurological deficits of mice [29]. In this study, TLR-4 inhibitor TAK-242 and NF-*κ*B inhibitor were used to treat MCAO-induced BV2 cells in vitro. Both inhibitors were found to inhibit proinflammatory expression and upregulate proinflammatory expression, similar to the effect of hesperidin, and mice treated with hesperidin in vivo could inhibit TLR-4 and p-NF-*κ*B expression levels. Therefore, the mechanism of hesperidin regulating phenotypic changes of MCAO-induced BV2 cells through TLR4-NF-*κ*B pathway was confirmed.

## 5. Conclusion

In conclusion, this study found that M1 microglia were overactivated in the infarct lateral brain tissue of MCAO mice, accompanied by overexpression of TLR4-NF-*κ*B in the inflammation-related pathway. And after the administration, hesperidin can improve the neurological deficit symptoms of MCAO mice, inhibit the expression of M1 proinflammatory related factors, and upregulate the expression of anti-inflammatory M2 molecules. In vitro experiments further showed that the microglial phenotype of MCAO-induced BV2 cells treated with TLR-4 inhibitor TAK-242 and NF-*κ*B inhibitor BAY 11-7082 was similar to that of hesperidin, verifying that hesperetin is neuroprotective by inhibiting TLR4-NF-*κ*B pathways, which provides new targets and strategies for neuroprotection and nerve repair after ischemic stroke.

## Figures and Tables

**Figure 1:** Hesperidin can improve the neural function defect with a protective role in MCAO mice. (a) Changes and comparison of neurological deficit scores of mice in MCAO and MCAO + hesperidin group 7 days after surgery. (b) Evaluation and statistics of cerebral infarct volume of mice in MCAO and MCAO + hesperidin group 7 days after surgery (*n* = 10). (c) Comparison and statistics of brain loss volume of mice in MCAO and MCAO + hesperidin groups 7 days after surgery. ^*∗*^*P* < 0.05, ^*∗∗*^ < .01, and ^*∗∗∗*^ < .001.

**Figure 2:** Expression of microglia-related molecules in infarcted lateral brain tissue of mice in MCAO group 7 days after surgery. (a–d) M1 microglia-related molecules of mice in sham, MCAO, and MCAO + hesperidin groups: mRNA expression levels of iNOS, CD11b, CD32, CD86, and comparative analysis. (e–h) Microglia-related molecules of mice in sham, MCAO, and MCAO + hesperidin groups: mRNA expression levels of CD206, Arg-1, TGF-*β*, and Ym1/2 and intragroup comparisons. ^*∗*^*P* < 0.05, ^*∗∗*^ < 0.01, and ^*∗∗∗*^ < 0.001.

**Figure 3:** Expression of microglia-related molecules and pathway proteins in infarcted lateral brain tissue of MCAO mice 7 days after surgery. (a, b) Expression levels of iba-1, iNOS, and Arg-1 of mice in sham, MCAO, and MCAO + hesperidin groups and statistical analysis. (c) Expression levels of p-NF-*κ*B and TLR-4 and statistical analysis mice in sham, MCAO, and MCAO + hesperidin groups. ^*∗*^*P* < 0.05, ^*∗∗*^ < 0.01, and ^*∗∗∗*^ < 0.001.

**Figure 4:** Levels of cytokines in the supernatant of cultured BV2 cells determined by ELISA. (a) TNF-*α* levels of the supernatant in normal group, MCAO group, MCAO + hesperidin (100 *μ*M) group, MCAO + TAK-242 group, and MCAO + BAY group. (b) IL-1*β* levels of the supernatant of BV2 cells in the above five groups. (c) TGF-*β* levels of the supernatant of BV2 cells in the above five groups. (d) IL-10 levels of the supernatant of BV2 cells in the above five groups. ^*∗*^*P* < 0.05, ^*∗∗*^ < 0.01, and ^*∗∗∗*^ < 0.001, and ns indicates no statistical significance.

**Figure 5:** Phenotypic changes and TLR4-NF-*κ*B expression levels of MCAO-induced BV2 cells in vitro. (a) Expression of iNOS, iba-1, Arg-1, TLR-4 and NF-*κ*B of BV2 cells in MCAO group, MCAO + hesperidin group, MCAO + TAK-242 group (TLR-4 inhibitor), and MCAO + BAY group (NF-*κ*B inhibitor). (b) Analysis of the expression levels of inos, iba-1, and Arg-1. (c) Statistical analysis of TLR-4 expression level of BV2 cells in MCAO group, MCAO + hesperidin group, MCAO + TAK-242 group (TLR-4 inhibitor), and MCAO + BAY group (NF-*κ*B inhibitor). (d) Statistical analysis of p-NF-*κ*B expression levels of BV2 cells in MCAO group, MCAO + hesperidin group, MCAO + TAK-242 group (TLR-4 inhibitor), and MCAO + BAY group (NF-*κ*B inhibitor). ^*∗*^*P* < 0.05 and ^*∗∗*^ < 0.01.

**Table 1:** Primer sequence.

Gene	Forward (5′ ⟶ 3′)	Reverse (5′ ⟶ 3′)
iNOS	CAAGCACCTTGGAAGAGGAG	AAGGCCAAACACAGCATACC
CD11b	CCAAGACGATCTCAGCATCA	TTCTGGCTTGCTGAATCCTT
CD32	AATCCTGCCGTTCCTACTGATC	GTGTCACCGTGTCTTCCTTGAG
CD86	TGATCGCCAACTTCAGTGAA	CAGAACACACACAACGGTCA
CD206	TGAGCTGTTTTGGTTGGGAC	CCCATCTGCAGTAACTGGTG
Arg-1	TCACCTGAGCTTTGATGTCG	CTGAAAGGAGCCCTGTCTTG
TGF-*β*	TGCGCTTGCAGAGATTAAAA	CGTCAAAAGACAGCCACTCA
Ym1/2	CAGGGTAATGAGTGGGTTGG	CACGGCACCTCCTAAATTGT
GAPDH	CGGAGTCAACGGATTTGGTCGTAT	AGCCTTCTCCATGGTGGTGAAGAC

## Data Availability

The datasets used and/or analyzed during the present study are available from the corresponding author upon reasonable request.
